# A Contrastive Predictive Coding-Based Classification Framework for Healthcare Sensor Data

**DOI:** 10.1155/2022/5649253

**Published:** 2022-03-15

**Authors:** Chaoxu Ren, Le Sun, Dandan Peng

**Affiliations:** ^1^Engineering Research Center of Digital Forensics, Ministry of Education, Nanjing University of Information Science and Technology, Nanjing, China; ^2^School of Computer Science and Network Engineering, Guangzhou University, Guangzhou, China

## Abstract

Supervised learning technologies have been used in medical-data classification to improve diagnosis efficiency and reduce human diagnosis errors. A large amount of manually annotated data are required for the fully supervised learning process. However, annotating data information will consume a large amount of manpower and resources. Self-supervised learning has great advantages in solving this problem. Self-supervised learning mainly uses pretext tasks to mine its own supervised information from large-scale unsupervised data. And this constructed supervised information is used to train the network to learn valuable representations for downstream tasks. This study designs a general and efficient model for the diagnosis and classification of medical sensor data based on contrastive predictive coding (CPC) in self-supervised learning, called TCC, which consists of two steps. The first step is to design a pretext task based on the idea of CPC, which aims to extract effective features between different categories using its encoder. The second step designs a downstream classification task with lower time and space complexity to perform a supervised type of training using the features extracted by the encoder of the pretext task. Finally, to demonstrate the performance of the proposed framework in this paper, we compare the proposed framework with recent state-of-the-art works. Experiments comparing the proposed framework with supervised learning are also set up under the condition of different proportions of labeled data.

## 1. Introduction

Healthcare as an important part of smart cities directly affects the quality of smart city construction. In recent years, the rapid growth of urban population density, population aging, and various chronic diseases have brought challenges to the development of smart healthcare [1]. This no longer meets the requirements of sustainable urban development, prompting a shift from hospital-centered to family-centered healthcare [2]. The application of various deep learning algorithms has made it less difficult to automatically classify diseases and has greatly improved the accuracy of disease classification [3, 4]. The classification model can be paired with various IoT devices for real-time diagnosis [5], and patients can grasp their health status at home without having to go to the hospital for checkups every time, which will ease the tension on medical resources and help the construction of smart medical care to achieve sustainable urban development.

However, traditional supervised learning training requires a large amount of labeled data to achieve good results. For medical data with few labels and a high labeling threshold [6], traditional supervised training is no longer suitable [7]. Self-supervised learning can well solve the problem of unlabeled medical data by creating pseudolabels [8]. Self-supervised learning methods learn more general features rather than task-specific features, so models using self-supervised learning can be reused for different tasks in the same domain and can better perform the task of classifying medical sensor data [9].

In this paper, we use contrastive predictive coding in self-supervised learning to accomplish the classification of medical sensor data. We build a **t**wo-step **C**PC-based **c**lassification framework (TCC) for medical sensor data and conduct experiments on two types of medical sensor data: electroencephalogram (EEG) and electrocardiogram (ECG). By establishing a model for real-time automatic classification, it helps to alleviate the increasing strain on medical resources and promote the sustainable development of smart cities.

In summary, the main contributions of this work are as follows.

We propose a two-step TCC model according to the architecture and ideas of contrastive predictive coding in self-supervised learning. First step, designing a contrastive predictive coding (CPC)-based pretext task for medical sensor data classification, then redesigning the arrangement of positive sample pairs and negative sample pairs. The second step is to design a lightweight and simple downstream classification model, which further improves the classification accuracy, achieving a very good result.

In order to verify that the pretext task is indeed learning useful features, we designed the classification experiments using fully supervised learning and the pretext task in the case of different numbers of sample labels (10%, 30%, 50%, 70%, and 100%). Experiments have proved that the pretext task is indeed learning useful features. When the number of sample labels is small, after using the CPC-based pretext task, the classification accuracy is still maintained at a very high level.

The rest of this paper is organized as follows: Section 2 introduces the related work, including two aspects; Section 3 presents TCC, which contains CPC-based pretext task (first step) and a downstream classification task (second step); Section 4 shows the experiment procedure and experiment results; and Section 5 concludes this paper and gives some future research directions.

## 2. Related Works

Many deep learning technologies have been applied to medical data classification and have achieved great success [10]. Automatic recognition of sleep classification through feature extraction started a long time ago [11]. Automatic classification of sleep states based on EEG has been a hot research topic in the field of health informatics.

### 2.1. Supervised Learning Classification Methods

Akara et al. [12] proposed a two-step training method to train their model, which is named DeepSleepNet. In their model, they utilized convolutional neural networks (CNN) to extract *z*-time-variable features and bidirectional-long short-term memory (Bi-LSTM) to learn transition rules among sleep stages automatically from EEG epochs. Sajad et al. [13] proposed a deep learning model called SleepEEGNet, which is composed of a convolutional neural network to capture time-variable features and frequency information. The model also used a sequence-to-sequence model to capture the complex and long short-term context dependencies between sleep epochs and scores. Huy et al. [14] proposed a hierarchical recurrent neural network named SeqSleepNet which treated the task as a sequence-to-sequence classification problem. Koushik et al. [15] performed end-to-end training on the EEG dataset using a time-distributed convolutional neural network.

### 2.2. Unsupervised Learning Classification Methods

Emadeldeen et al. [16] proposed a model based on unsupervised learning named TS-TCC and designed contrastive learning through weak data augmentation and strong data augmentation. A cross-view prediction task is one of the highlights of this paper. Hogeon et al. [17] proposed a model named IITNet which \hl{utilized} residual neural networks and bidirectional-long short-term memory networks for sleep classification. Mohsenvand et al. [18] extended the SimCLR [19] framework to time-series data and realized different classification tasks. Yang et al. [20] proposed a self-supervised learning model called ContraWR and conducted experiments on three EEG datasets. Zhang et al. [21] proposed a generative adversarial network-based data enhancement method to improve accuracy and prevent overfitting.

## 3. TCC Framework

### 3.1. Contrastive Predictive Coding

Contrastive predictive coding was proposed in 2018. The purpose is to predict future features from past features by training a neural network, which can be used on pictures or data with time-series features. The core idea of this method is contrastive learning. We can learn more global and meaningful structures instead of small irrelevant details by predicting far into the future. The core of contrastive learning is to learn a mapping function *f* and encode the sample *x* into its representation f(x). The core of contrastive learning is to make this $f$ satisfy the following formula:

(1) $$\begin{array}{c} s\left(f\left(x\right),f\left(x^{+}\right)\right)\gg s\left(f\left(x\right),f\left(x^{-}\right)\right).\; \end{array}$$

Here x^+^ is a sample similar to *x*, and x^−^ is a sample that is not similar to *x*. s() is a function that measures the degree of similarity between samples. A typical score function is the vector inner product. That is to optimize the following expectations:

(2) $$\begin{array}{c} E_{x,x^{+},x^{-}}\left[-\text{log}\left(\frac{e^{f{\left(x\right)}^{T}f\left(x^{+}\right)}}{e^{f{\left(x\right)}^{T}f\left(x^{+}\right)}+e^{f{\left(x\right)}^{T}f\left(x^{-}\right)}}\right)\right]. \end{array}$$

Contrastive predictive coding is an approach for unsupervised learning from high-dimensional data by translating a generative modeling problem to a classification problem. The contrastive loss, or InfoNCE loss, in CPC, inspired by noise contrastive estimation (NCE) [22], uses cross-entropy loss to measure how well the model can classify the “future” representation amongst a set of unrelated “negative” samples. Such design is partially motivated by the fact that the unimodal loss like MSE has not had enough capacity but learning a full generative model could be too expensive. The (3) represents the mutual information between *x* and *c* that we want to maximize, where *c* is the potential content representation vector and *x* is the sample. By doing so, we extract the underlying latent variables that the inputs have in common.

(3) $$\begin{array}{c} I\left(x;c\right)=\sum_{x,c}p\left(x,c\right)\text{log}\frac{p\left(x,c\right)}{p\left(x\right)}. \end{array}$$

For EEG signals, we have made a little innovation here, which is to predict by establishing positive and negative sample pairs instead of predicting the future. For positive sample pairs, they belong to the same category, and the features extracted by train data should be used for prediction. It is highly similar to the coding features of waiting train data. For negative sample pairs, because they belong to different categories, when predicting the features extracted by train data, the less similar the coding features of the waiting train data, the better. So, the goal is to maximize the similarity between positive sample pairs and minimize the similarity between negative sample pairs.

We establish positive and negative sample pairs, where the positive sample pair contains 8 different samples belonging to the same category, and the four left and four right of the negative sample pair belong to the same category, but the left and right are different categories. The label of the positive sample pair is 1, and the label of the negative sample pair is 0. The left half of the training sample is called the training set, and the right half is called the waiting training set.  Figure 1 describes the details. Algorithm 1 describes the process to establish positive sample pairs and negative sample pairs.

### 3.2. Pretext Task

The structure of the pretext task model is shown in Figure 2. Giving a batch of train set samples *x*^*t*^ and a batch of waiting train set samples *x*^*w*^, an encoder *g*_*enc*_ maps the input into *Z*_*j*_^*T*^ (0 ≤ *j* ≤ *t*), *Z*_*j*_^*W*^ (0 ≤ *j* ≤ *t*), respectively. Next, a GRU model *g*_*ar*_ summarizes all *Z*_*j*_^*T*^(0 ≤ *j* ≤ *t*) in the latent space and produces a context latent representation *c*. Finally, we use the content vector *c* for multistep prediction and calculate the loss value with *Z*_*j*_^*W*^ (0 ≤ *j* ≤ *t*). The loss function uses binary_crossentropy, the formula is as follows:

(4) $$\begin{array}{c} L_{\text{pre}}=-\frac{1}{N}\overset{N}{\underset{i=1}{\sum }}y_{i}\cdot \text{ log}\left(p\left(y_{i}\right)\right)+\left(1-y_{i}\right)\cdot \text{ log}\left(1-p\left(y_{i}\right)\right), \end{array}$$

where*y* is the true label (1 for positive sample pairs and 0 for negative sample pairs) and p(y) is the calculated probability of being a positive sample.

The encoder part contains four identical blocks, and each block contains a dense layer, a batch normalization layer, an activation layer, and finally a dense layer to output the coding features. It is worth noting that the quality of the pretext task training directly affects the performance of the downstream classification model, so the model of the pretext task needs to be fully trained. Here we have trained 20 epochs. At the same time, since the training samples are randomly selected, in order to ensure the probability of the samples being selected, each epoch is trained thousands of times to ensure that the pretext task can be fully trained.

### 3.3. Classification Task

The downstream classification task uses the encoder part of the pretext task. The encoder part saves the model parameters after the pretext task is trained and loads the model parameters directly. The classification model structure is shown in Figure 3. We can see that the model is very lightweight and concise, and no particularly complex structure is used. The classification model contains two Conv1 layers that are not exactly the same; they have different filters and kernel size.

In order to maintain the dimensionality of the input data of the encoder layer, a sample is copied four times before classification. For example, for a sample *x*_1_, the shape of its input model should be [*x*_1,_*x*_1,_*x*_1,_*x*_1_]. In order to speed up the convergence of the model and get good results, monitor the change of the validation set loss. When the performance is not improved within two epochs, the learning rate will be reduced to 1/3 of the original, and the initial learning rate is set to 0.001. The loss function here uses categorical_crossentropy, which is used as a loss function for multiclass classification models where there are two or more output labels. The output label is assigned a one-hot category encoding value in the form of 0 and 1. Algorithm 2 describes the overall classification model.

## 4. Experiments and Results

### 4.1. Datasets

The American Academy of Sleep Medicine (AASM) divides sleep data into five stages, namely awake (W), stages 1–3 (N1, N2, and N3), and rapid eye movement (REM) [23]. In addition, N1, N2, and N3, respectively, represent transitional sleep, light sleep, and deep sleep, respectively. We aim to classify the input EEG signal into one of five classes and download the sleep-EDF dataset from the PhysioBank. The sleep-EDF database contains 197 whole-night polysomnographic(PSG) sleep recordings, containing EEG, EOG, chin EMG, and event markers, where we used a single EEG channel (Fpz-Cz) with a sampling rate of 100 Hz [24].  Table 1 shows the total number for each class.  Figure 4 shows the waveform variations for each category.

### 4.2. Pretext Task Results

Figure 4 shows the trend of the accuracy of the training set and test set in the pretext task. It can be seen from Figure 5 that the result of the training set is more than 99%, and the result of the test set is more than 98%. If the pretext task is not fully trained, the accuracy of the downstream classification task is about 70%.

### 4.3. Classification Task Results

Table 2 shows the confusion matrix after inputting all the datasets into the classification model. The last three columns represent the performance indicators of each category according to the confusion matrix. It can be seen that the classification effect for all sleep stages is very good, especially the N1 category, which shows a good classification effect compared to other models [12, 13], which shows that our pretext task is quite effective. The average value of F1 is 88.09, and the overall accuracy is 88.70. We compare the performance using two metrics namely the accuracy (ACC) and the macro-averaged F1-score (MF1), with other proposed models.  Table 3 shows the details.

### 4.4. Few Data Results

Inspired by [25], we did this experiment.  Figure 6 shows the change trend of the accuracy of the classification model prediction when the pretext task is used and the supervised learning is used when samples of different proportions are used. The supervised learning here refers to the model without using the encoder part parameters saved by the pretext task, directly use the encoder part for training. The results show that when the number of sample labels is small, the accuracy of the model can still be maintained at a high level after using the pretext task.

### 4.5. Experiment: Sustainability of CPC-Based Model

This experiment validates the sustainability of the model on another dataset: the MIT-BIH supraventricular arrhythmia database (MIT-BIH-SUP). This dataset includes 78 half-hour ECG recordings chosen to supplement the examples of supraventricular arrhythmias in the MIT-BIH arrhythmia database [26]. The Association for Advancement of Medical Instrumentation (AAMI) classifies the heartbeats of arrhythmia patients into five classes: normal beat (N), supraventricular ectopic beat (S), ventricular ectopic beat (V), fusion beat (F), and unclassifiable beat (Q) [27]. Since the number of F and *Q* data is very small, we use this model to perform three classification experiments on N, S, and V. We resample the sampling rate from 128 Hz to 251 Hz and divide the dataset into a training set and test set according to the ratio of 9 : 1 and the results are shown in Table 4. The accuracy of the deep learning model proposed in [28] is only 88.2%. In contrast, TCC has a huge improvement.

### 4.6. An Industry Application of TCC for Improving the Development of Sustainable Smart Cities

Among all the facilities provided by smart cities to citizens, smart medical treatment is the most important and most concerned about the well-being of the people. Smart medical combines intelligent technology with medical health and can use a variety of wearable devices to obtain human health data. Doctors, researchers, and healthcare professionals can analyze these data to obtain better-personalized diagnoses and solutions. By deploying the classification model on small mobile devices and cooperating with the use of various sensors, patients can master their health status in real-time, avoiding the various complicated steps of going to the hospital every time, which is conducive to the construction of a sustainable smart city.  Figure 6 shows an industry application of TCC for sustainable smart cities.

Patients can select appropriate medical monitoring equipment according to their actual situation. This equipment will transfer the obtained medical sensor data to the TCC system, and the system will analyze whether the medical data is abnormal in real-time. In the event of an abnormality, a warning will be issued to prompt the patient to go to the hospital on time, and the abnormal medical data flow will be recorded to facilitate the doctor's diagnosis and analysis.

## 5. Conclusion

We exploit a self-supervised deep learning framework for sleep stage classification. Based on the architecture and ideas of contrastive predictive coding, this paper proposes a CPC-based pretext task that uses positive sample pairs and negative sample pairs to design contrastive learning, and the model finally extracts different types of effective features. Using the encoder part of the pretext task, a very lightweight classification model is designed, which achieves very good results on the dataset. The F_1_-scores of classifying awake, N1, N2, N3, and, REM sleep stages are 90.09%, 84.65%, 89.81%, 90.58%, and 85.30%, respectively. At the same time, we verified that in the case of a small amount of data labels, the model still achieved good results, and the performance of the model exceeded the supervised learning. We extend the experiments in another dataset, which shows the robustness and sustainability of the model more efficiently. In the future, we plan to use more complex or time-based classification models to further improve the accuracy of model classification. Although the sample imbalance did not affect the final experimental results, we still plan to utilize some machine learning methods, such as the synthetic minority oversampling technique to solve this problem.

## Figures and Tables

**Figure 1:** The division method of the positive sample pair, the negative sample pair, and the training set to be trained. Looking from the top down, the top half and the bottom half are positive and negative sample pairs, respectively. Viewed from left to right, the left half is the training set, and the right half is the waiting training set.

**Figure 2:** Model architecture.

**Figure 3:** Waveform diagram for each category.

**Figure 4:** Pretext task training results.

**Figure 5:** The change trend of the accuracy of different numbers of samples in different models.

**Figure 6:** An industry application of TCC for sustainable smart cities.

**Algorithm 1:** Establish sample pairs.

**Algorithm 2:** Overall classification model.

**Table 1:** The sleep-EDF dataset.

	Awake	N1	N2	N3	REM	Total
Total number	8285	2804	17799	5703	7717	42308

**Table 2:** Confusion matrix and various evaluation indicators.

	Awake	N1	N2	N3	REM	PR (%)	RE (%)	F_1_ (%)
Awake	7270	235	349	79	352	92.55	87.75	90.09
N1	55	2572	75	4	98	78.58	91.73	84.65
N2	278	269	15418	396	1438	93.25	86.62	89.81
N3	69	2	506	5126	0	91.29	89.88	90.58
REM	183	195	186	10	7143	79.09	92.56	85.30
Macro avg								88.09
ACC	88.70%							

**Table 3:** Comparison between our proposed model against others.

	ACC (%)	MF1 (%)
SSL-ECG [9]	74.58	65.44
SimCLR [9]	78.91	68.60
TS-TCC [9]	83.00	73.57
DeepSleepNet [6]	82.00	76.88
IITNet [10]	84.00	77.70
SleepEEGNet [7]	84.26	79.66
CPC-based (ours)	88.70	88.09

**Table 4:** Confusion matrix and various evaluation indicators.

ACC (%)	N(%)			S(%)			V(%)		
	PR	RE	F_1_	PR	RE	F_1_	PR	RE	F_1_
97.30	97.90	99.42	98.65	89.80	77.28	83.07	95.24	87.65	91.29

## Data Availability

The labeled datasets used to support the findings of this study are available from the corresponding author upon request.
